# Maternal Resilience and Postpartum Depression at the Neonatal Intensive Care Unit

**DOI:** 10.3389/fped.2022.864373

**Published:** 2022-05-10

**Authors:** Eva Mautner, Christina Stern, Alexander Avian, Maria Deutsch, Herbert Fluhr, Elfriede Greimel

**Affiliations:** ^1^Division of Obstetrics, Department of Obstetrics and Gynecology, Medical University of Graz, Graz, Austria; ^2^Department of Medical Psychology and Psychotherapy, Medical University of Graz, Graz, Austria; ^3^Institute for Medical Informatics, Statistics and Documentation, Medical University of Graz, Graz, Austria

**Keywords:** neonatal intensive care unit, depression, resilience, postpartum, maternal, depressive symptoms, women, mothers

## Abstract

**Background:**

The neonatal intensive care unit causes maternal stress and postpartum depressive symptoms in preterm and term mothers. Personal resources like maternal resilience are usually not considered in counselling these women.

**Objective:**

This study aims to evaluate the resilience and differences in postpartum depression after admission of newborns at the neonatal intensive care unit.

**Methods:**

This prospective pilot study was conducted in a single teaching hospital in Austria from December 2016 until December 2018. Sixty women completed two internationally validated questionnaires, the Edinburgh Postnatal Depression Scale (EPDS) to evaluate depressive symptoms and the Resilience Scale RS-13 to measure maternal resilience during the postpartum period (3 to 10 days postpartum). Additionally, women answered two open questions about burdens and relief.

**Results:**

Twenty women (34%) showed lower resilience scores. The 39 high-resilient women (66%) showed significantly less depression (*p* = 0.005). Women reported social support from their partner (*n* = 15), health professionals and psychologists (*n* = 15), family and friends (*n* = 12), and child-specific relief, e.g., spending time with the newborn and involvement in care (*n* = 7) as the most helpful variable during the first postpartum period.

**Conclusion:**

The experience of having a newborn at the neonatal intensive care unit is a challenging event for women. Women have different resilience parameters. Mothers with lower resilience will benefit from social support and emotional health-promoting activities.

## Introduction

Depressive disorders occur frequently during pregnancy and the postnatal period (1). The predicted prevalence of postpartum depression (PPD) varies from 6.5 to 15 percent during the first year (1–4). In clinical practice and research, PPD is defined, if inconsistently, as depression that occurs within 4 weeks after childbirth up to 1 year (2). Symptoms comprise excessive worrying, tearfulness, feelings of inadequacy, loss of appetite, insomnia, and depressed mood. PPD is distinct from “maternity blues,” which includes symptoms that appear and disappear within the first days after delivery (5).

Mothers of infants born prematurely show high PPD rates (20-40%), primarily in the early postnatal period (6–8). One recent meta-analysis found evidence of a higher probability of PPD up to 24 weeks after childbirth (4). Preterm birth has become increasingly common because of medical improvements in neonatal intensive care and advanced treatment of high-risk pregnancies (9). The global figure for the preterm rate is approximated at 10.6% (uncertainty interval 9.0-12.0) (10).

However, it has been found that the NICU environment causes similar distress in term mothers (11). Both newborns and parents are exposed to different stressors in the hospital intensive care environment (7, 12).

Several studies have concentrated on resilience as a protective individual resource regarding depression (13–15) or found a negative correlation with depression (16). The term resilience is applied to different phenomena varying from prevention of mental health disturbance to effective adaptation and recovery after life adversities (13). Resilience includes the capacity to tolerate major stress and accept adjustment in life and may contain post-traumatic personal growth (13, 14). It includes the ability to bounce back from severe adverse experiences by staying open and developing tactics that result in an enhanced quality of life (14, 15, 17, 18). Wagnild and Young suggested “a two-dimensional structure of resilience” originated from two aspects “acceptance of self and life” and “personal competence” (16). Three helpful domains were recognised to improve resilience after exposure to difficult situations. These domains are secure attachment, positive emotions, and a purpose in life (13). Generally, research proposes that resilience is a modifiable construct and not an inherent trait of individuals and can be learned (13–15).

The objective of the current survey was to examine differences in depression of women showing high or lower resilience scores after the admission of their newborns at the NICU. Additionally, we investigated burdens and relief in two open questions. We hypothesised that highly resilient women show less depression.

## Methods

This prospective questionnaire pilot study was carried out in a single teaching hospital tertiary referral centre for obstetrics and gynaecology in Europe/Austria. After the purpose of the study was explained, women received the informed consent forms and the German questionnaire battery. The minimum to maximum time interval from birth to study inclusion was 3 to 10 days postpartum. The study protocol was approved by the local ethics committee (Nr.: 28-269 ex 15/16).

### Participants

Eligible patients were recruited for this survey. Inclusion criteria were mothers with preterm or term births (23 + 0 to 42 weeks of gestation) who were separated from their newborns because of intensive care treatment at the neonatal ward. Exclusion criteria were parents' psychiatric illness and/or drug abuse, and the inability to understand German.

### Measures

Two questionnaires were used, the Edinburgh Postnatal Depression Scale (EPDS) to detect depression (19) and the Resilience Scale (RS-13) to measure resilience.

The EPDS is a reliable, internationally applied, and well-validated screening device to detect postnatal depression. The German translation of the EPDS showed satisfactory internal consistency reliability (Chronbach's alpha = 0.82). A cut-off value of 10/11 is recommended for Austrian women (20). According to Muzik et al., it appeared to yield maximal sensitivity (0.87) and specificity (0.87) in detecting major depression in an Austrian population (20).

The RS-13 is the short German version of the RS-25 scale by Wagnild and Young (16). The German version has two subscales “personal competence” and “acceptance of self and life.” It was validated by Leppert et al.. We used the general score, which ranges from 13 to 91. Higher values signify higher resilience (above or equal to 72); values lower than 72 lower resilience (lower than 72) “The internal consistency of the variables of the German RS-13 was acceptable (Chronbach's alpha = 0.90). The retest reliability was 0.62 (21).”

To specify what was distressing and helpful for women after the newborns' admission to the NICU, two open questions administered burdens (“What did you find distressing?”) and relief (“What did you find helpful?”) were asked. Additionally, single Likert scales were used to measure prospectively the amount of anxiety, perceived postnatal stress, and general psychological distress. Women evaluated the degree of anxiety and postnatal stress throughout the early preterm period on a scale from 0 (not at all) to 100 (very much). General psychological distress was established with a single Likert scale from 0 (not at all) to 5 (most experienced distress).

A demographic and medical data sheet completed the questionnaire with maternal characteristics: age, gravidity, number of children alive, mode of delivery, weight of the newborns, gestational week at birth, maternal hospitalisation before birth, education level, living situation, employment status, and financial situation.

### Statistical Analysis

Data are displayed as mean and standard deviation or median and interquartile range (IQR) for continuous variables. Categorical data are shown as absolute and relative frequencies. Differences between the two resilience groups were investigated using the Mann-Whitney *U*-test or the *T*-test for continuous data and Fischer's exact test or χ^2^-Test for categorical data. A value *p* < 0.05 was considered statistically significant. Statistical analyses were performed using IBM SPSS 24.0 (IBM Corp., Armonik, NY, USA).

## Results

Sixty women were included. One woman dropped out because she forgot to answer the resilience questions. Therefore, complete data sets were available for 59. All newborns had to be treated at the NICU for a variety of reasons, such as preterm labour (*n* = 17), complicated twin pregnancies (*n* = 12), complications after maternal pre-eclampsia or HELLP-Syndrome (*n* = 8), perinatal infections (*n* = 9), infant respiratory distress syndrome (*n* = 5), fetal bradycardia (*n* = 2) and others (6), e.g., fetal hydronephrosis or fetal anal atresia.

As shown in Table 1, demographic characteristics did not differ between the resilience groups in gravidity, mode of delivery, weight of the newborns, gestational week at birth, living situation, hospitalisation before birth, employment status, and financial situation. However, we found statistically significant differences in age. Highly resilient women were significantly younger than older ones (*p* = 0.018).

**Table 1:** Clinical and demographic characteristics by level of resilience.

	**Low resilience <72 (*n* = 20)**	**High resilience ≥72 (*n* = 39)**	
	***M*** **±** ***SD Median (IQR) N (%)***	***M*** **±*****SD Median (IQR) N (%)***	***P***
Age (M ± SD)	34 ± 5	30 ± 5	0.018^*^
Gravidity	2 (1, 2)	1 (1, 2)	0.233
Mode of delivery			0.442
Elective primary caesarean	7 (36.8%)	20 (51.3%)	
Emergency caesarean	6 (31.6%)	7 (17.9%)	
Spontaneous vaginal	6 (31.6%)	12 (30.8%)	
Weight of the newborns (Median ± SD*)*	2357 ± 1037	1959 ± 996	0.161
Gestational week at birth	34 (33-40)	33 (30-38)	0.157
Living situation			0.655
With children	1 (5.0%)	1 (2.6%)	
With partner and children	12 (60.0%)	21 (53.8%)	
With partner, children and Grandparents	3 (15.0%)	4 (10.3%)	
With partner	4 (20.0%)	13 (33.3%)	
Hospitalization before birth (Median, IQR days)	11 (3–20)	4 (1–28)	0.445
Employment status			0.724
Not employed	2 (10%)	5 (12.8)	
Full-time employed	11 (55.0%)	24 (61.5%)	
Part-time employed	7 (35.0%)	10 (25.6%)	
Financial situation			0.637
Very satisfied	3 (15.0%)	9 (23.1%)	
Satisfied	15 (75.0%)	28 (71.8%)	
Less satisfied	2 (10.0%)	2 (5.1%)	

* *significant difference between the groups*.

In the whole study population (not in the Tables), women had on average 1.4 children (range from 1 to 4 children). The level of education was evaluated at four levels: primary (*n* = 3, 5%), secondary (*n* = 17, 28.3%), higher education (*n* = 19, 31.7%) and university (*n* = 21, 35%). The current relationship was described as living with partner (*n* = 17, 28.3%), with partner and children (*n* = 34, 56.7%), with partner, children, and grandparents (*n* = 7, 11.7%) and as single mother/ woman with children (*n* = 2, 3.3%), respectively. The employment status of the whole study sample before pregnancy was full-time employed (*n* = 36, 60%), part-time employed (*n* = 17, 28.3%), and not employed (*n* = 7, 11.7%). Most of the women were either very satisfied (*n* = 12, 20%) or satisfied (*n* = 44, 73.3%) with their financial situation.

### Main Results for Resilience and Depression

Thirty-nine women (66.1 %) of the whole study population experienced themselves as highly resilient, 20 women (33.9%) demonstrated lower resilience scores. As shown in Table 2, women with high resilience showed significantly lower depression scores as measured by the EPDS compared to women with lower resilience (*p* = 0.005). The mean depression score of women with lower resilience (*N* = 39, *M* = 13, SD = 6) was above the cut-off value of 10 for an Austrian population, indicating more depression compared to women with high resilience (*N* = 20, *M* = 9, SD = 6).

**Table 2:** Differences in the EPDS, perceived stress, anxiety, and general psychological distress by level of resilience.

	**Low resilience (*n* = 20)**	**High resilience (*n* = 39)**	
	***M*** **±** ***SD Median (IQR)***	***M*** **±*****SD Median (IQR)***	***P***
Depression	13 ± 6	9 ± 6	0.005
Perceived stress	70 (50-80)	70 (40-80)	0.532
Anxiety	80 (40-90)	70 (50-80)	0.519
General psychological Distress	3 (2–4)	3 (2–4)	0.451

Twenty-nine women made one or more comments regarding specific burdens and relief during the last few days after admission of their newborns to the neonatal ward. Most of these women expressed worries about the state of health of the child and/or the uncertain situation or found the separation from the child distressing. Seven women expressed helplessness (see all statements in Table 3):

**Table 3:** Burdens and relief at the NICU during the first 10 days.

What did you find distressing? (46 comments from 29 women)	• Burdens Worries about the state of health of the child and/or the uncertain situation (*n* = 16) Separation from the child (*n* = 9) Helplessness (*n* = 7) Worries about not being a good mother (*n* = 3) Uselessness (*n* = 3) Commuting to the hospital (*n* = 3) Providing milk/pumping (*n* = 2) Concern about another child (*n* = 1) Mood swings (*n* = 1) Emptiness (*n* = 1)
What did you find helpful? (63 comments from 28 women)	• Social Support (45 comments) Support from the partner (*n* = 15) Support from family and friends (*n* = 12) Support form health professionals (*n* = 15) Support from other patients (*n* = 3) • Child specific resources/relief (18 comments) Spending time with the newborn/involvement in care (*n* = 7) Confidence in the caretaker and that the baby is doing well (*n* = 6) Perception of a stable health status and progression of the newborn (*n* = 5)

*n = based on number of comment*.

Twenty-eight women responded with one or more comments regarding experienced relief. Two categories were found: firstly, social support (45 comments) and secondly, child-specific relief/resources (18 comments, see Table 3). One woman expressed a sense of meaning or meaningfulness due to the new situation.

## Discussion

One-third of the whole study population showed lower resilience scores and as expected, those women had significantly higher depressive scores measured with the EPDS. Several studies found higher prevalence of postpartum depression among women with hospitalised newborns at the NICU, especially in preterm infants (4, 6, 7, 9). McGowan et al. declared that mothers felt little support at the NICU, showed lower emotional willingness for discharge, lower family support, and diminished awareness of the newborn and her own well-being (7). Additional studies found that symptoms of anxiety and depression were common among all parents in the NICU (22). However, from a perspective of resources, parents of very-low-birth-weight infants were more hopeful than the general population (23).

Women in our study pilot population showed several maternal resources in stressful situations. Of the study population, 66.1% showed high resilience during their time at the NICU. Remarkably, medical characteristics, such as the weight of the newborns, gestational week at birth, gravidity, and mode of delivery or hospitalisation before birth, were not associated with higher or lower resilience. As literature confirmed, resilience indicates inner strength, optimism, competence, flexibility, and the ability to function effectively when faced with adversity (13, 16). Younger women showed even higher resilience scores than older ones. There are no references for this result. We assume that these women had the best ability to cope with the life event of having a baby in the NICU, including the capacity to tolerate major stress and accept change (13, 14). This needs further examination.

As we did not find differences in perceived stress and high or lower resilience scores, we suggest that women generally face acute stress in the NICU environment, but find different ways to recover. In prior studies, the most stressful situations were the newborn appearance, changes in the parental role, worries about developmental difficulties, and sights and sounds of the NICU environment (7, 11). Acute stress can be measured easily with single Likert scales, which might be an uncomplicated way to evaluate the functioning of preterm mothers during the first postpartum period.

Our results suggest that at the NICU, social support may have an essential role in coping with maternal stress, reducing depressive symptoms and improving resilience. The most important factor was social support from the partner, family members and friends but also social support from health care providers, such as getting information, and involvement in care and emotional and practical support. The need to involve mothers and parents empathetically from the beginning of their child's stay at the NICU was also suggested in other studies (24). Women learn to handle the situation through guidance from nurses and paediatricians in understanding their newborn and learning how to support their baby during their stay at the NICU. The experience of the growing capacity to manage and cope with the NICU situation increases resilience and decreases NICU-related stress, depressive feelings of helplessness, and inadequacy. Women learn to live with what is beyond their control and find meaning in redefining their priorities to become advocates for their newborns.

Enhancing the ability to experience positive emotions was mentioned as an important building block of resilience (13). Positive interactions in daily life with health professionals may boost positive emotions, such as being smiled at when interacting with the newborn at the NICU.

Resilience training courses are not often established among adults. In a systematic review, Leppin et al. evaluated the efficacy of resilience training programs and found a moderate effect of generalised stress-directed programs on enhancing resilience. They also found that trauma-induced stress-directed programs significantly improved stress and depression (25).

As we confirmed an association between depression and resilience, the treatment of depression seems to be another step in improving resilience. There are several recommendations considering the treatment of PPD (1–3, 26, 27). First line interventions for mild and moderate symptoms of depression include psychosocial interventions that improve support, such as peer support and nondirective counselling. Additionally, formal time-limited psychotherapy or psychological treatment that addresses the challenges of the transition to motherhood is advised (2). Psychological care and communication about the health situation of the newborns, fears, needs, and resources are easy to administer and most helpful in getting more competence and improving resilience.

### Strengths and Limitations

In our study, we used an internationally validated depression screening instrument whose diagnostic performance has been good in other studies (1); this can be seen as a strength of the study, since the EPDS is specific for the evaluation of depression in postpartum women in our local population. We measured depressive symptoms once in our study population. However, women had the choice to get psychological support immediately after the survey. One element to discuss is the influence of maternal socio-economic status on our results. As the socio-economic level was high in the whole study population, most of the women had undergone higher education (31.7%) or had a university degree (35%) and were very satisfied (20%) and satisfied (73.3%) with their financial situation. Another one is the single-centre pilot study design with small numbers, which might affect the generalizability of the study to the general population or other countries. However, this was a very specific group of women with newborns at the NICU. Lower socio-economic levels could have an influence on resilience and depression rates. This could be clarified in further international studies.

## Implications for Clinical Practice

One third of our study population showed lower resilience scores, which was connected with more depressive symptoms. For clinical practice, our results highlight the significance of being able to identify women with lower resilience who cannot cope as easily with the experience of the hospitalisation of their newborns at the NICU. Social support from the partner, friends and family as well as from health professionals during the time at the NICU seems to play an important role in improving resilience. Providing opportunities for women to understand, manage, care for and monitor their newborns during hospitalisation increases parental feelings of self-confidence and competence. Especially women with lower resilience will benefit from emotional health-promoting activities and stress-directed programs to develop better strategies regarding resilience parameters, “personal competence” and “acceptance of self and life” (16, 21).

## Data Availability Statement

The raw data supporting the conclusions of this article will be made available by the authors, without undue reservation.

## Ethics Statement

The studies involving human participants were reviewed and approved by Ethikkommission der Medizinischen Universität Graz. The patients/participants provided their written informed consent to participate in this study.

## Author Contributions

EM, MD, EG, and AA contributed substantially to conception and design, acquisition of data, and analysis and interpretation of data. EM, MD, EG, AA, CS, and HF contributed to drafting the article and revising it critically for important intellectual content and gave final approval for the version to be submitted. All authors contributed to the article and approved the submitted version.

## Conflict of Interest

The authors declare that the research was conducted in the absence of any commercial or financial relationships that could be construed as a potential conflict of interest.

## Publisher's Note

All claims expressed in this article are solely those of the authors and do not necessarily represent those of their affiliated organizations, or those of the publisher, the editors and the reviewers. Any product that may be evaluated in this article, or claim that may be made by its manufacturer, is not guaranteed or endorsed by the publisher.
